# A 2015 outbreak of flea-borne rickettsiosis in San Gabriel Valley, Los Angeles County, California

**DOI:** 10.1371/journal.pntd.0006385

**Published:** 2018-04-20

**Authors:** Kimberly Nelson, Alice N. Maina, Angela Brisco, Chelsea Foo, Curtis Croker, Van Ngo, Rachel Civen, Allen L. Richards, Kenn Fujioka, J. Wakoli Wekesa

**Affiliations:** 1 San Gabriel Valley Mosquito and Vector Control District, West Covina, California, United States of America; 2 Viral and Rickettsial Diseases Department, Naval Medical Research Center, Silver Spring, Maryland, United States of America; 3 Acute Communicable Disease Control, Los Angeles County Department of Public Health, Los Angeles, California, United States of America; 4 CDC/CSTE Applied Epidemiology Fellowship Program, Centers for Disease Control and Prevention, Atlanta, Georgia, United States of America; 5 Community Health Services Program, Los Angeles County Department of Public Health, Los Angeles, California, United States of America; UTMB, UNITED STATES

## Abstract

Although flea-borne rickettsiosis is endemic in Los Angeles County, outbreaks are rare. In the spring of 2015 three human cases of flea-borne rickettsiosis among residents of a mobile home community (MHC) prompted an investigation. Fleas were ubiquitous in common areas due to presence of flea-infested opossums and overabundant outdoor cats and dogs. The MHC was summarily abated in June 2015, and within five months, flea control and removal of animals significantly reduced the flea population. Two additional epidemiologically-linked human cases of flea-borne rickettsiosis detected at the MHC were suspected to have occurred before control efforts began. Molecular testing of 106 individual and 85 pooled cat fleas, blood and ear tissue samples from three opossums and thirteen feral cats using PCR amplification and DNA sequencing detected rickettsial DNA in 18.8% of the fleas. Seventeen percent of these cat fleas tested positive for *R*. *felis*-specific DNA compared to under two (<2) percent for *Candidatus* R. senegalensis-specific DNA. In addition, serological testing of 13 cats using a group-specific IgG-ELISA detected antibodies against typhus group rickettsiae and spotted fever group rickettsiae in six (46.2%) and one (7.7%) cat, respectively. These results indicate that cats and their fleas may have played an active role in the epidemiology of the typhus group and/or spotted fever group rickettsial disease(s) in this outbreak.

## Author summary

Outbreaks of flea-borne rickettsiosis are rare despite the endemic status in Los Angeles County. In the spring of 2015 three human cases of flea-borne rickettsiosis among residents of a mobile home community (MHC) prompted an investigation. Fleas were found in all common areas at the MHC due to presence of flea-infested opossums and overabundant outdoor cats and dogs. The MHC was summarily abated in June 2015, and within five months, flea control and removal of animals significantly reduced the flea population. Two additional epidemiologically-linked human cases detected at the MHC were considered to have occurred before control efforts began. Molecular testing of cat fleas, immunological testing of opossums and feral cats collected at the site indicated active transmission of flea-borne rickettsiosis. This study represents the first flea-borne rickettsial outbreak that summary abatement approach was used to reduce its intensity.

## Introduction

Acute febrile flea-borne rickettsial diseases are caused by intracellular gram-negative bacteria *Rickettsia typhi* and *Rickettsia felis*, which are known to be transmitted to humans by the bite of *Xenopsylla cheopis* (oriental rat flea) and *Ctenocephalides felis* (cat flea); both fleas are found on many domestic and peri-domestic vertebrate hosts [1]. In recent years, additional flea transmitted *Rickettsia* has been identified in fleas and their hosts, both living in close proximity to people, warranting such rickettsial infections in humans referred to as flea-borne rickettsiosis. Unfortunately, when rickettsial infections are detected in humans the clinical diagnostic tests almost never distinguish between rickettsial species–*R*. *typhi* (typhus group—TG) or *R*. *felis* (spotted fever group- SFG) [2]. The commonly reported flea-borne rickettsiosis in humans is murine typhus whose known causative agent is *R*. *typhi*. Commercially available clinical serological diagnostic tests commonly show cross-reactivity among the pathogens in the TG and SFG. Confirmation of these infections requires positive serology in paired acute and convalescent serum samples of a four-fold or greater change in immunoglobulin G (IgG) and M (IgM)-specific antibody titer reactive to *R*. *typhi* or other *Rickettsia* species antigen by indirect immunofluorescence assay (IFA). In most clinical settings, rarely are paired acute and convalescent serum samples collected, and California Department of Public Health resolved this shortcoming through special guidelines that achieved confirmation of murine typhus serologically or by nucleic amplification in a single serum specimen of elevated IgG and IgM antibody reactive to *R*. *typhi* or other *Rickettsia* species by IFA or DNA amplification, respectively (CDPH 2011) [3]. Consequently, laboratory confirmation of murine typhus may not represent true cases, but cases of flea-borne rickettsiosis. Although these cases are reported as murine typhus without identifying the actual rickettsial pathogen but for purposes of consistent reporting they are reported as murine typhus. Here we identify such cases as flea-borne rickettsiosis and attempt to determine the responsible rickettsial agent for the current outbreak.

On average, there are more than 200 human cases of murine typhus reported in the United States each year. This disease is not nationally reportable, so the true number of cases is unknown [4]. In areas where this disease is endemic (California, Hawai’i, and Texas), providers and clinical laboratories are mandated to report cases to their local public health departments [2,5]. In California, most of the flea-borne rickettsial disease cases occur in Los Angeles and Orange counties, but concentrated outbreaks of the disease are rare [2]. Prior to 2015, the last documented cluster of human flea-borne rickettsial disease in Los Angeles County occurred in 2009 [6,7]. Over the past decade, the incidence of flea-borne rickettsial disease in Los Angeles County (LAC) has increased. In 2014, 51 cases were reported statewide [44 (86%) in LAC], 88 cases [69 (78%) in LAC] in 2015, and 90 cases [70 (78%) in LAC] in 2016. These cases in LAC occur in suburban communities through interactions between wildlife, domestic animals, and humans.

Since the initial discovery of *R*. *felis* in *C*. *felis* in 1990 [8,9,10], the association of *R*. *felis* with *C*. *felis* has been well-documented and the connection between zoonotic diseases and free-roaming animals has become an issue [8,9,10,11,7]. The last two decades have witnessed an increase in the recognition of new *R*. *felis*-like organisms (RFLOs), particularly *Rickettsia asembonensis* and *Candidatus* Rickettsia senegalensis, whose distributions and host ranges appear to mimic those of *R*. *felis* [12]. Although there are no studies published concerning its ability to cause clinical illness, *R*. *asembonensis* was recently detected in the blood of monkeys (*Macaca fascicularis*) in Malaysia [13], and in dogs’ blood in South Africa [14]. Another agent with close genetic composition to *Ca*. R. senegalensis was detected in the blood of febrile patients from Senegal [15].

Free-roaming animals have increasingly become a source of flea-borne infectious diseases that are controlled in domestic cat populations through routine veterinary care and flea control. When this care is lacking, the consequence is increased potential health risks for other domestic animals and humans [11]. Incidental infection transfer also occurs when free-roaming animals are fed outdoors. Wildlife, free-roaming cats, and domestic animals are brought in proximity when food is left outdoors, increasing the potential for exchanging fleas. When ectoparasites of wildlife become too numerous, they infest new hosts, increasing the risk that they may transmit disease to domestic animals and humans [16,17].

Three human case reports of flea-borne rickettsiosis among residents of a single 95-unit mobile home community (MHC), with disease onsets from April 23rd to June 9th, 2015 prompted an initial investigation, and subsequent abatement order by the San Gabriel Valley Mosquito and Vector Control District (District) [18]. The Los Angeles County Department of Public Health (LACDPH) initiated active case finding to look for additional outbreak-associated cases during this time period and helped to coordinate a multi-agency notification, and abatement in the MHC [19,4]. The District conducted the abatement order in the MHC and coordinated overall surveillance, control, and mitigation efforts [20]. Here we discuss the outbreak, samples collected to identify the etiological agent(s), and efforts made to mitigate the risk factors to public health.

## Materials and methods

The San Gabriel Valley Mosquito and Vector Control District (District) is located in Los Angeles County, California. It includes more than 54,000 hectares of Los Angeles County and is bordered to the north by the San Gabriel Mountains where a plethora of wild animals exist. From April to June 2015, the District received reports from LACDPH of three active cases of flea-borne typhus in its jurisdiction from a 95-unit MHC. The cases were investigated to determine the environmental conditions supporting this outbreak and necessary efforts to prevent its recurrence.

### Human cases

In April 2015, case A from the MHC was hospitalized for four nights and case B was hospitalized for six nights (Table 1). In June, case C from the same MHC was hospitalized for five nights [4]. A hospital infection preventionist reported the cases to LACDPH and they were forwarded to LACDPH Environmental Health Department and the District. From April to June 2015, LACDPH conducted enhanced case finding for *Rickettsia typhi*-positive (Quest Diagnostic, Inc.; IFA test) cases at all acute care facilities and local clinics within the catchment area of the MHC. Outbreak-associated cases were defined as MHC residents with symptom onset of fever with headache or rash from March 1^st^, 2015 through August 31^st^ 2015, and/or positive *R*. *typhi* or *R*. *rickettsii* laboratory test (immunoglobulin M (IgM) >1:128 and/or immunoglobulin G (IgG) >1:128. Additional criteria include elevated liver function tests (ALT or AST), decreased platelet counts, and proximity in time and space for epidemiological-linkage to the outbreak. Cases A, B, and C were initially tested by Quest Diagnostics, Inc (San Juan Capistrano, CA) and two additional cases were tested and confirmed via indirect fluorescent antibody assays (IFA) by LAC Public Health Laboratory (part of LACDPH). Paired acute and convalescent specimens of the cases were not available. Unlike LACDPH Laboratory, it’s not common practice for clinical commercial tests to include a full rickettsial panel of *R*. *typhi* and *R*. *rickettsii*. The State of California Department of Public Health guidelines interprets the detection of elevated IgG and IgM antibody reactive to *R*. *typhi* or other *Rickettsia* species antigen by IFA titer of ≥ 128 in a single serum specimen in addition to having specified clinical symptoms as confirmed cases [3]. These cases were part of anonymized LA County public health surveillance data.

**Table 1:** Case characteristics of five flea-borne rickettsiosis cases residing in the investigated mobile home community in Los Angeles County, California during the outbreak period of March 1^st^ through August 31^st^, 2015.

Case	Age	Sex	Cat Owner	Dog Owner	Onset Date	Fever	Headache	Rash	Hospitalized	Hosp Nights	ALT (U/L)	AST (U/L)	Platelets (K/mm^3^)	*R*. *typhi*		*R*. *rickettsii*	
														IgG	IgM	IgG	IgM
**A**	42	F	No	Yes	4/9/15	Yes	Yes	No	Yes	4	92	84	72	1:128	≥1:256	ND	ND
**B**	51	M	Yes	Yes	4/20/15	Yes	Yes	No	Yes	6	57	120	56	<64	1:64	ND	ND
**C**	67	F	Yes	Yes	6/5/15	Yes	Yes	No	Yes	5	189	140	119	1:128	1:128	ND	ND
**D**	48	F	No	Yes	Unsp*	No	Yes	Yes	No	0	ND	ND	ND	1:128	<64	1:64	<64
**E**	47	F	No	Yes	8/20/15	Yes	Yes	Yes	No	0	ND	ND	ND	1:64	<64	1:128	<64

* Denotes unspecified indicating that other ongoing health conditions made it difficult to assess a true onset date for flea-borne rickettsial infection.

### Environmental investigation

The initial investigation began in June 2015 with a survey of the property which included counting and photographing the number of pets and animals outdoors, the number of outdoor feeding sources (water bowls and food), the presence and locations of free roaming animals, available harborage, and the presence of uncovered garbage bins. A door to door inspection and discussion with the residents of this MHC was conducted to inform them of the outbreak and symptoms of rickettsial disease, and the association of fleas and illnesses in the community. Discussions regarding appropriate cause of action were conducted between LACDPH, Environmental Health, and District staff. Opossums in the neighborhood were trapped using two live traps (Tomahawk Live Trap, Tomahawk, WI) set on selected properties in the MHC. Fleas were combed off the opossums trapped, identified to species level [21], and tested by species-specific molecular methods for presence of rickettsial pathogens.

A summary abatement order was issued by the District to the MHC on June 24, 2015 to clean up the property. Specific requests included removal of animal feces, enforcement of MHC property rules limiting the pets to one animal per property, and regular flea control to reduce the population of fleas. The order also mandated that MHC residents cease outdoor feeding of pets and contract a pest control company to reduce the number of feral animals on the property. In addition, the property manager notified residents to provide flea control for all animals under their care, those tenants with more than one pet against the MHC homeowner rules and regulations to give them up and register their “single animal pet” with the property manager. This directive was necessary because most tenants had more pet animals some up to 32, contrary to their property lease contracts.

On August 24, 2015 a multi-agency community event was held at a shopping center adjacent to the MHC by LACDPH, the District, the state Senator’s office District 20, the city, and other regulatory agencies, to discuss public health risk posed by flea-borne rickettsiosis and encourage residents of the MHC to participate in reducing this risk. Residents of the MHC with symptoms of flea-borne rickettsial disease per case definition within the past three months were encouraged to provide blood samples for testing at no cost to them. Five individuals participated in the blood draw event and their blood tested by commercially available IFA tests, two of them were positive and was considered epidemiologically-linked human cases from this MHC. The tests were performed by Quest Diagnostics and/or confirmed by LAC Public Health Laboratory using commercially available FDA-approved IFA clinical tests.

The property owner contracted with two pest control companies, one to control fleas and the other to remove feral animals on the property. The numbers of outdoor feeding sources were recorded monthly to determine the effectiveness of the property owners’ efforts. Flea control was conducted every 14 days, and the population of fleas was monitored bi-weekly by placing six 16 cm x 11 cm glue boards (PIC Corporation, Linden, NJ) throughout the property. Fleas collected on glue boards were counted and averaged by month to assess flea control efforts. Free-roaming domestic animals were counted monthly during morning walks of the property to monitor the impact of vertebrate/animal trapping efforts. A regression analysis (JMP v 10/0: http://www.jmp.com) was used to calculate the coefficient of determination (static) which correlated control measures conducted at the MHC against the number of outdoor wildlife, feeding sources, and flea activity. Fleas, blood, and ear tissue samples were retrieved from all cats removed by the vertebrate trapper and the opossums by the District from the MHC (13 cats, and 3 opossums) for epidemiologic studies. One rat retrieved from the trap was dead and no flea, blood, or ear tissue samples were collected for testing. The Naval Medical Research Center tested all samples collected from the MHC epidemiologic study to determine the prevalence of rickettsial agents responsible for the outbreak.

### Molecular and serological testing

Fleas combed off animals trapped at the MHC were washed in molecular grade water and mechanically disrupted with disposable pellet pestles (Fisher Scientific, Pittsburgh, PA). Genomic DNA was extracted with Prepman Ultra sample preparation kits (Applied Biosystems, Foster City, CA). Genomic DNA from cat and opossum ear tissues and blood clots were extracted using the DNeasy blood and tissue kit (QIAGEN, Valencia, CA) according to the manufacturer’s instructions with a final elution volume of 50 μl.

All fleas from cats (n = 46) and 20 fleas from each opossum (n = 60) were processed individually. Remaining fleas from the three opossums were processed in pools of 18–20 fleas (n = 1,553). Flea DNA, and DNA from the cat and opossum blood and tissues were initially screened for rickettsial DNA using a genus-specific quantitative real-time PCR (qPCR) assay (Rick17b) targeting the 17-kDa antigen gene [22]. DNA from the individual flea, cat, and opossum blood, and tissue samples that tested positive by the Rick17b assay were subsequently tested using a group-specific qPCR assay (RfelB) [23] and three species-specific assays, namely, (1) *R*. *felis* specific assay (Rfel_phosp_MB) that targets the membrane phosphatase gene from *R*. *felis* [24], (2) the *R*. *typhi* species specific qPCR assay (Rtyph) which targets a fragment of the *R*. *typhi ompB* gene [23], and (3) the *Rickettsia asembonensis*-specific qPCR assay (Rasem), which targets a fragment of *R*. *asembonensis ompB* gene [25,26]. Similarly, the DNA from the pooled fleas was screened using the Rick17b, Rtyph, and the Rasem qPCR assays.

PCR amplification and sequencing of *gltA* was attempted for a subset of 7 individual flea DNA including one DNA sample that was positive for rickettsial DNA using the Rick17b qPCR assay but negative for *R*. *felis* DNA based on the Rfel_phosp_MB qPCR assay, 2 samples that had discordant cycle threshold (Ct) values between Rick17b qPCR and Rfel phosp_MB qPCR assays and 4 flea DNA samples positive with both the Rick17b and the Rfel_phosp_MB qPCR assays to confirm the specificity of Rfel_phosp_MB. PCR amplification of *gltA* gene was attempted for all ear tissue DNA that tested positive for rickettsia DNA by qPCR, as previously described [20]. Sequencing reactions were performed in the forward and reverse directions utilizing the Big Dye Terminator v3.1 Reaction Cycle sequencing kit (Life Technologies, Carlsbad, CA) according to the manufacturer’s instructions using an ABI 3500 genetic analyzer (Applied Biosystems). Sequence assembly was performed using CodonCode Aligner version 5.0.1 (CodonCode Corporation, Centerville, MA). Blast searches were performed in NCBI websites.

Evidence of previous infection of animals with spotted fever group (SFGR) and typhus group (TGR) rickettsiae was assessed using group-specific immunoglobulin G (IgG) enzyme-linked immunosorbent assays (ELISAs) as previously described [25,27,28], using *R*. *typhi* str. Wilmington and *R*. *conorii* str. Morocco as the TGR and SFGR ELISA antigens, respectively. Serum samples were diluted 1:100 and screened for antibodies against rickettsiae using both the SFGR and TGR ELISAs. Screen positive samples (those with net absorbance of ≥ 0.5) were titered by 4-fold serial dilution (100–6,400). Commercial anti-cat IgG (KPL, Gaithersburg, MD) and anti-opossum IgG (Alpha Diagnostics Intl. Woodlake Center, San Antonio, TX) antibodies labeled with horseradish peroxidase (HRP) were used in both ELISAs.

Ethics Statement: The San Gabriel Valley Mosquito and Vector Control District (SGVMVCD) do not have a formal Institutional Animal Care and Use Committee (IACUC) since it is not considered a research institution. However, it does follow the protocols for animal handling for disease surveillance purposes as outlined by the California Department of Public Health, Vector Borne Disease Section, and adhered to American Veterinary Medical Association (2013) guidelines for animal euthanasia. SGVMVCD as a cooperative member of Mosquito and Vector Control Association of California is exempt from requirement of holding a scientific permit under FG code 1002, 4005, and 4011 of the California Department of Fish and Wildlife (CDFW) to collect and sample small mammals for disease surveillance purposes.

## Results

### Human cases

Initially, three human (A, B, and C) cases were identified from the MHC with illness onset ranging from April to June 2015. The LACDPH active case finding reported two additional epidemiologically-linked (D and E) cases of the outbreak for the period from March 1^st^ through August 31^st^ 2015 (Table 1). They were predominantly female (4/5) their ages ranged from 42 to 67 years; all were dog owners and two also owned cats. All experienced headaches, three had fever (A, B, and C), and two (D and E) had a rash. The first three (A, B and C) cases were hospitalized for a total of 15 days (mean 5); the remaining two cases were discovered from on-site blood draw at the community event (D and E). The same three cases (A, B, and C) showed lower platelet count and elevated liver function enzymes (ALT and AST). All cases recovered without complication. All five cases had antibodies reactive to *R*. *typhi* or other *Rickettsia* antigens with titers ≥ 1:128 via IFA testing except case B which together with cases C and D are considered epidemiologically-linked and part of the outbreak (Table 1).

### Environmental investigation

Two live traps set in June 2015 on the selected plots at the MHC yielded two opossums infested with 615, and 1,087 cat fleas, respectively. Another opossum was trapped in September and was infested with 487 cat fleas. Flea control was conducted at the MHC every 14 days beginning in September 2015 by a professional pest control company. To assess its effectiveness, glue boards strategically distributed in the MHC at six locations were retrieved every two weeks from September to November. The glue boards placed on location prior to treatment contained as many as 39 fleas. The number of fleas on the glue boards declined significantly after the first treatment (n = 36, r² = 0.5813, p≤ 0.05), and the trend continued over time (number of months), until no fleas were collected for two consecutive collection sessions (Fig 1).

**Fig 1:** Average number of fleas (plus standard error) collected on glue boards (n = 36) from Sep to Nov 2015 at the mobile home community in San Gabriel Valley, California.

The MHC hired a wildlife trapper to remove outdoor vertebrate pests from the MHC. Thirteen cats were removed by the trapper from September to November. The number of fleas on the cats removed from the MHC declined over time (n = 13, r² = 0.7512, p < 0.05) with the first cat collected in September having 13 fleas on it, and the one collected in November having no fleas. Subsequently, the number of cats outdoors from June through November also significantly declined from 29 to 4 (n = 87, r² = 0.914, p < 0.05) over time (Fig 2).

**Fig 2:** Abundance of outdoor wildlife and outdoor feeding sources from Jun to Nov 2015 at the mobile home community in San Gabriel Valley, California.

The number of outdoor feeding stations at the MHC also decreased significantly (n = 90, r² = 0.9697, p < 0.05; Fig 2). The decline in the population of fleas on the ground and on cats, free-roaming animals, and wildlife, and the decreased prevalence of outdoor feeding ultimately decreased the risk at the MHC of acquiring flea-borne typhus.

### Molecular and serological testing

A total of 13 cats and three opossums were trapped around the MHC over the study period. Pooled fleas (n = 1,553) combed from these animals were screened for rickettsiae with the genus specific qPCR assay (Rick17b), *R*. *typhi* specific qPCR assay, and *R*. *asembonensis*- specific qPCR assay. Eighty-five pools were tested, with 74 (85.33%) testing positive for rickettsiae (Table 2). Further screening was qPCR assay negative for both *R*. *typhi* and *R*. *asembonensis*.

**Table 2:** Summary of *Rickettsia* genus-specific qPCR assay (Rick17b) assessment of *Ctenocephalides felis* pools (n ≤ 20 individual fleas/pool) from 3 opossums at the mobile home community in Los Angeles County, California.

Opossum (n = 3) Identification Number#	Total # of Fleas	Total # of Pools Tested	Total # of Pools Rick17b qPCR Positive	% Rick17bpositive	MIR
1	119	10	10	100	8.4
2	967	52	51	97.87	5.3
3	467	23	13	56.52	2.8
Total	1553	85	74	85.33	4.8

One hundred and six individual fleas from cats and opossums were tested. From 9 of 13 cats, 46 fleas, and from three opossums, 60 fleas making a total of 106 fleas were tested for rickettsial DNA (Table 3). Twenty of these fleas (18.8%) were positive for *Rickettsia* DNA using the genus-specific assay Rick17b. Of these, 18 were positive for *R*. *felis* using the Rfel_phosp_MB assay. None of the fleas were positive for *R*. *typhi* or *R*. *asembonensis*-specific qPCR assays.

**Table 3:** Summary of qPCR assay results for individual fleas from 3 opossums and 13 cats at the mobile home community in Los Angeles County, California.

	Total # of animals	# of fleas	# of fleas tested	#*Rickettsia* genus-specific Rick71b positive (%)	*R*. *felis*-specific Rfel_phosp_MB positive (%)	*R*. *typhi*-specific Rtyph positive (%)	*Ca*. R. senegalensis-sequence positive (%)	# of Positive animals (%)	MIR
Opossums	3	2189	60	9 (15)	8 (13.33)	0	1 (1.66)	3 (100)	4.1
Cats	13	46	46	11 (23.91)	10 (21.73)	0	1 (2.17)	9 (69.23)	23.9
Total	16	2235	106	20 (18.8)	19 (16.9)	0	2 (1.88)	12 (75)	8.9

To confirm the identity of rickettsiae identified by the qPCR assays, PCR amplification and sequencing of the *gltA* gene was done in a subset of seven individual flea DNA preparations. Seven 1186-bp *gltA* sequences were generated, of which five were 100% identical to each other and to *R*. *felis* URRWXCal2 (Accession no. CP000053). The five samples included four that had tested positive for both Rick17b and Rfel_phosp_MB, and one of the two samples that had discordant Ct. The remaining two sequences were 100% identical to each other and to *Candidatus* Rickettsia senegalensis (Accession number KF666472), and included one that was positive for Rick17b but negative for Rfel_phosp_MB, assay, and one that had discordant Ct values.

A total of 13 cat sera and three opossum sera were assessed for antibodies against TGR and SFGR by ELISA and the presence of *Rickettsia* DNA by qPCR assays. Of the sera tested for the presence of SFGR- and TGR-specific IgG, 6/13 (46.15%) had IgG antibodies reactive against TGR antigens with endpoint titers ranging from 1600 to 6400 (Table 4). One of the 13 cat sera (7.69%) was positive for antibodies against SFGR antigens with an endpoint titer of 100. None of the opossum sera were positive for antibodies against SFGR- or TGR-specific IgG.

**Table 4:** Summary of percent (%) prevalence of IgG antibodies in 3 opossums and 13 cat sera from animals collected at the mobile home community in Los Angeles County, California.

	Total #	SFG Screen	SFG Titer	TG Screen	TG Titer	Overall Prevalence
Opossums	3	0	0	0	0	0
Cats	13	1 (7.69)*	100	6 (46.15)	≥ 1600	6 (46.15)

* One cat serum sample was positive for SFG and TG IgG ELISA at titers of 6400 and 100, respectively.

The blood clots and tissues from 13 cats and 3 opossums were also assessed for the presence of *Rickettsia* DNA. All blood clot DNA preparations from cats and opossums were negative for *Rickettsia* DNA whereas three of thirteen cat tissues tested positive for *Rickettsia* DNA (Rick 17b with Ct values > 35). One of three cat tissue DNA preparations tested positive for *R*. *felis* by group-specific qPCR RfelB assay, but all three cat tissue preparations were negative for other PCR assays and none produced amplicons for sequencing.

## Discussion

An outbreak of five cases of flea-borne rickettsial disease occurred at the MHC within the District. It is highly likely that additional infections occurred due to the abundance of fleas on the property, but went undetected due to a mild presentation and/or lack of testing.

The etiologic agent of flea-borne rickettsial diseases has been debated for years. *R*. *typhi* has been known historically as the etiologic agent of murine typhus [29,1,30,2]. There were three hospitalized and two non-hospitalized epidemiologically-linked cases at the MHC that had *R*. *typhi* or other *Rickettsia* antibody titers ≥ 1:128 except one of hospitalized cases with titers ≥ 1:64 via IFA test, all in private clinical laboratory or/and LAC Public Health Laboratory. Although human testing met state guidelines the only limitation of the clinical diagnostic testing of all five cases was the use of a single serological sample instead of the paired acute and convalescent samples. Such samples were not available because it is uncommon for clinicians to collect paired samples from patients in clinical settings. Physicians often overlook rickettsial infections and by the time such tests are deemed necessary for patient care a dose of antibiotics/chemotherapy would have been administered rendering collection of paired serological sample impossible. The clinical IFA test conducted on single patient sera does not confirm murine typhus but confirms rickettsial infection either of TG or SFG. The epidemiology of rickettsial diseases in southern California, and especially San Gabriel Valley in Los Angeles County show that *R*. *typhi* is the predominant human *Rickettsia* pathogen compared to SFG-transmitted *R*. *rickettsii*, thus it has not been important from a public health standpoint to differentiate between TG and SGF infections [2,4]. Current assays examining IgG/IgM titers with indirect fluorescent antibody assays do not always differentiate between antibodies against *R*. *typhi* and other *Rickettsia* species, and the former is assumed to be the etiologic agent for murine typhus, therefore of flea-borne rickettsiosis [31]. A more accurate differentiation between *R*. *typhi* and other *Rickettsia species* could be made through PCR based assays if a blood specimen could have been available from acute symptomatic individuals. Unfortunately, at the time of investigation, acute blood specimens from the three hospitalized cases were unavailable.

Samples from the animals and fleas removed from the MHC were tested for the presence of the different etiologic agents. *Rickettsia felis* was detected in fleas obtained from animals at the MHC, which supports prior research that elevated the potential role of *R*. *felis* previously referred to as ELB as an etiological agent of flea-borne rickettsial disease in relation to *R*. *typhi*, and implicated opossums and rodents as the main hosts [2,32,33]. However, results showed that both *R*. *felis* and *Ca*. R. senegalensis were present in cat fleas, although the association of *R*. *felis* with human disease seems poor [34]. The focus was on *R*. *typhi* where 46.15% of cat sera removed from the MHC were positive, and none of the opossum blood had any rickettsial DNA. Low level IgG-positive opossum and lack of rickettsial DNA in opossums aligns with findings from previous studies [12,34]. Alternatively, the presence of antibodies against *R*. *typhi* in cats suggests that it could still be active within the peri-domestic and domestic animal community and this may suggest that cats provide another mechanism for maintaining typhus in southern California. Furthermore, *R*. *typhi* was not detected in the cat fleas, which corroborates past findings [35] that *R*. *typhi* may still be present in the environment at a very low but infectious level and/or possibly carried by another flea species and hosted by other mammals beside opossum and cats.

Beside *R*. *felis*, the present study detected *Ca*. R. senegalensis in cat fleas. This corroborates the findings of two previous studies that reported existence of the “RFLO” in southern California [12,35]. Although the previous studies reported *R*. *asembonensis* at a relatively low rate (0.3% of 597 fleas tested) in the same region [12], the present study did not confirm that finding. Although two RFLOs have been detected in the blood of dogs, monkeys, and humans [15,13,14], their ability to cause disease in mammalian species has not yet been proven. The relationship (symbiosis, mutualism, or parasitism) between the host and the rickettsiae has not been elucidated for any of the RFLOs. It has been suggested that all rickettsiae can potentially be pathogenic to vertebrate hosts [36]. This is evidenced by the findings that *R*. *slovaca*, *R*. *helvetica* and *R*. *parkeri* tick endosymbionts were associated with human disease years after they were discovered [37,38,39].

Within five months of focused abatement implementing mitigation measures, the potential risk of rickettsial and other flea-borne diseases infection was reduced based on several observations within the neighborhood under investigation. The achievement of mitigation measures involved flea control, trapping and removal of feral cats, and opossums, providing flea-collars to residents for cats and dogs, and removal of outdoor feeding sources by the property owner and tenants. The role of public health agencies was education and coordination, and that of vector control was identifying the responsible parties–property owner and tenants–and ensuring they contracted with professional pest control whose work was certified at completion. More importantly no additional cases of flea-borne rickettsioses were detected. Ultimately, the success of this approach as spearheaded by public health agencies was measured by the absence of new cases of flea-borne typhus, but the MHC must continue to adhere to its policies to ensure that public health risk previously present do not re-occur.
